The article "Pemetrexed Induces S-Phase Arrest and Apoptosis via a Deregulated Activation of Akt Signaling Pathway" was retracted in 2024. Reasons: duplicated images; duplicated data; duplicate publication; overlap with earlier publications.

# Pemetrexed Induces S-Phase Arrest and Apoptosis via a Deregulated Activation of Akt Signaling Pathway

**DOI:** 10.1371/journal.pone.0097888

**Published:** 2014-05-21

**Authors:** Kun-Chieh Chen, Tsung-Ying Yang, Chun-Chi Wu, Chi-Chih Cheng, Shih-Lan Hsu, Hsiao-Wen Hung, Jian-Wei Chen, Gee-Chen Chang

**Affiliations:** 1 Division of Chest Medicine, Department of Internal Medicine, Taichung Veterans General Hospital, Taichung, Taiwan, Republic of China; 2 Institute of Biomedical Science, National Chung Hsing University, Taichung, Taiwan, Republic of China; 3 Institute of Medicine, Chung Shang Medical University, Taichung, Taiwan, Republic of China; 4 Department of Medical Research, Chung-Shan Medical University Hospital, Taichung, Taiwan, Republic of China; 5 Department of Education and Research, Taichung Veterans General Hospital, Taichung, Taiwan, Republic of China; 6 Department of Life Sciences, National Chung Hsing University, Taichung, Taiwan, Republic of China; 7 Department of Medicine, School of Medicine, National Yang-Ming University, Taipei, Taiwan, Republic of China; University of Pecs Medical School, Hungary

## Abstract

Pemetrexed is approved for first-line and maintenance treatment of patients with advanced or metastatic non-small-cell lung cancer (NSCLC). The protein kinase Akt/protein kinase B is a well-known regulator of cell survival which is activated by pemetrexed, but its role in pemetrexed-mediated cell death and its molecular mechanisms are unclear. This study showed that stimulation with pemetrexed induced S-phase arrest and cell apoptosis and a parallel increase in sustained Akt phosphorylation and nuclear accumulation in the NSCLC A549 cell line. Inhibition of Akt expression by Akt specific siRNA blocked S-phase arrest and protected cells from apoptosis, indicating an unexpected proapoptotic role of Akt in the pemetrexed-mediated toxicity. Treatment of A549 cells with pharmacological inhibitors of phosphatidylinositol 3-kinase (PI_3_K), wortmannin and Ly294002, similarly inhibited pemetrexed-induced S-phase arrest and apoptosis and Akt phosphorylation, indicating that PI_3_K is an upstream mediator of Akt and is involved in pemetrexed-mediated cell death. Previously, we identified cyclin A-associated cyclin-dependent kinase 2 (Cdk2) as the principal kinase that was required for pemetrexed-induced S-phase arrest and apoptosis. The current study showed that inhibition of Akt function and expression by pharmacological inhibitors as well as Akt siRNA drastically inhibited cyclin A/Cdk2 activation. These pemetrexed-mediated biological and molecular events were also observed in a H1299 cell line. Overall, our results indicate that, in contrast to its normal prosurvival role, the activated Akt plays a proapoptotic role in pemetrexed-mediated S-phase arrest and cell death through a mechanism that involves Cdk2/cyclin A activation.

The article "Pemetrexed Induces S-Phase Arrest and Apoptosis via a Deregulated Activation of Akt Signaling Pathway" was retracted in 2024. Reasons: duplicated images; duplicated data; duplicate publication; overlap with earlier publications.

## Introduction

In Taiwan, lung cancer is the leading cause of cancer death and it causes more than 8,500 deaths per year [1]. More than half the patients diagnosed with lung cancer present with metastatic disease. Non-small-cell lung cancer (NSCLC) accounted for more than 85% of all lung cancer. The median survival is only 4–6 months for advanced or metastatic NSCLC patients when untreated [2]. Systemic chemotherapy provides survival benefit and relieves cancer-related symptoms for these patients. Platinum-based (cisplatin or carboplatin) doublets are the standard treatment for these patients with good performance status. Despite recent advances in the treatment, with the number of attractive treatment options for patients with NSCLC increasing, the five-year survival rate is only about 13–20% [2], [3].

The concept of maintenance therapy in lung cancer has stirred a great deal of interest over the last decade. Several randomized studies have been conducted to find out the usefulness of maintenance therapies for advanced NSCLC [4]. Pemetrexed, a compound that belongs to the family of thymidylate synthase inhibitors, has been widely used in cancer chemotherapy. Pemetrexed is currently used in combination with cisplatin for first line treatment of advanced NSCLC and malignant pleural mesothelioma. Pemetrexed in combination with cisplatin provided better efficacy than other doublet chemotherapy and attractive tolerability in treatment of nonsquamous NSCLC. In addition, pemetrexed maintenance therapy may further extend progression free survival and overall survival in these patients [5].

The presumed mode of action of pemetrexed is to halt DNA replication through its effects on cellular deoxynucleotide pools; collisions of DNA replication forks with these complexes convert them into DNA double-strand breaks (DSBs), subsequent induction of S-phase growth arrest, and potentially lethal lesions that may trigger apoptosis [6]. Pemetrexed has demonstrated broad antitumor activity against several types of human cancer cells, including NSCLC [7]–[9], and is clinically used as a maintenance therapy after cisplatin-based doublet chemotherapy in advanced NSCLC [9]. Understanding the mechanisms underlying the antitumour properties of pemetrexed is needed for optimization of therapeutic targeting by pemetrexed. To date, however, the targets and anticancer mechanisms of this compound remain largely unclear.

The oncoprotein Akt (also known as protein kinase B, PKB) is recognized to be a primary mediator of the downstream effects of phosphatidylinositol 3-kinase (PI_3_K), coordinating a variety of intracellular signals and, thus, controlling cell responses to extrinsic stimuli, regulating cell proliferation and survival, and promotes cell surviva and proliferation [10]. Increased Akt activation is a hallmark of diverse neoplasias providing both proliferative and antiapoptotic survival signals [11]–[14]. Although the role of the PI_3_K/Akt pathway in cell survival is well established, there are some exceptions where PI_3_K and Akt are obviously involved in promotion of cell death [15]–[18]. Recent studies have shown that Akt/PKB is activated by DNA damaging agents [19]. These findings raise the possibility that Akt may be activated by pemetrexed during DNA damage. A previous report demonstrated that pemetrexed induced the activation of the PI_3_K/Akt pathway, which is inhibited by a specific PI_3_K inhibitor, Ly294002 [20]. However, the role of Akt activation in pemetrexed-mediated cellular and molecular events and its mechanisms are unclear. Our previous report demonstrated that pemetrexed induced S-phase arrest and apoptosis of human NSCLC A549 cells via both ERK-CDK2/cyclin A and ataxia telangiectasia mutated (ATM)-p53 activation pathways [21], [22]. The present study was undertaken to determine: 1) whether pemetrexed activates Akt in human NSCLC A549 cells; 2) the role of Akt activation in pemetrexed-mediated growth arrest and cell death; and 3) whether activation of Akt plays a role in pemetrexed-induced growth arrest and apoptotic cell death, and, if so, by what mechanisms. Surprisingly, we found that prolonged Akt activation caused by pemetrexed treatment resulted in increased Cdk2/cyclin A activity leading to cell cycle arrest and apoptosis.

The article "Pemetrexed Induces S-Phase Arrest and Apoptosis via a Deregulated Activation of Akt Signaling Pathway" was retracted in 2024. Reasons: duplicated images; duplicated data; duplicate publication; overlap with earlier publications.

## Materials and Methods

### Reagents

Pemetrexed (Alimta) was obtained commercially from Lilly Research Laboratories (Eli Lilly, Indianapolis, IN, USA) and dissolved in sterile distilled water at a stock concentration of 1 mM. Anti-phospho-Akt^S473^ (#4060), Wortmannin (#9951), and 2-(4-morpholinyl)-8-phenyl-4H-1-benzopyran-4-1 (Ly294002) (#9901) were purchased from Cell Signaling Technology (Danvers, MA., USA). Anti-β-actin (sc-47778), anti-Cdk2 (sc-6248), anti-Cyclin A (sc-751), anti-Cyclin E (sc-198), anti-GSK3β sc-81462) anti-phospho-GSK3β (sc-81494), Akt siRNA (sc-29195) were purchased from Santa Cruz (Santa Cruz, CA., USA). Propidium iodide (PI) was obtained from Sigma Chemical Company (St. Louis,Mo., USA). Hoechst 33342 (#H1399) was obtained from Invitrogen Detection Technologies (Eugene, Oregon, USA). A terminal deoxynucleotidyl transferase-mediated dUTP-fluorescinnick end-labeling (TUNEL) assay kit was purchased from Life Technology (#23210) (Carlsbad, CA., USA). Anti-phospho-Histone H1 (#06-570) was purchased from Merck Millipore (Billerica, MA., USA).

### Cell culture

Human lung cancer A549 and H1299 cells were obtained from American Type Culture Collection (ATCC; Manassas, VA., USA). Both cell lines were cultured in RPMI 1640 supplemented with 5% fetal bovine serum, 2 mM glutamine, and antibiotics (100 unit/ml penicillin and 100 µg/ml streptomycin), at 37°C in a 5% CO_2_ humidified atmosphere. Culture medium was changed every two days.

### Determination of cell cycle distribution

Cells were treated with pemetrexed, and then trypsinized and washed with phosphate-buffered saline (PBS), and fixed in 75% ethanol at 4°C for 30 min. The fixed cells were washed with PBS and incubated with 100 µg/ml RNase A and propidium iodide (40 µg/ml) at 37°C for 30 min. Cells were collected and analyzed by a flow cytometer (Becton Dickinson, Mountain View, CA, USA). Cell cycle distribution was analyzed using Cell-FIT software (Becton Dickinson, Mountain View, CA, USA).

### Protein preparation and western blotting analysis

Cells were cultured without or with pemetrexed for indicated time periods. Cell lysate was extracted as described elsewhere [21]. Protein content was determined by the Bradford method. For western blot analysis, equal amounts of protein samples were separated by sodium dodecylsulphate-polyacrylamide gel electrophoresis (SDS-PAGE) and blotted onto PVDF membrane, and then blocked with Tris-buffered saline with 0.1% Tween-20 and 5% non-fat dry milk at room temperature for 1 h. Primary antibody was used to react with the blots at 4°C overnight, and then the blots were incubated with horseradish peroxidase-labeled secondary antibody. Immunoreactive bands were visualized using a Western Lightning Chemiluminescence kit (Perkin Elmer LAS, Inc. Waltham, MA., USA). To confirm specific effects on activation of the Akt, total cell lysates were separated by SDS-PAGE and subjected to western blotting the transferred membrane was blocked with 1% of BSA for 1 h followed by adding anti-phospho-Akt-Ser^473^ antibody 4°C overnight, and then the blots were incubated with horseradish peroxidase-labeled secondary antibody in 1% of BSA. Immunoreactive bands were visualized using Western Lightning Chemiluminescence kit (Perkin Elmer LAS, Inc. Waltham, MA., USA).

### Apoptotic cell determination

Cells were washed with cold PBS. Apoptotic cells were determined by a terminal transferase-mediated dUTP fluorescein nick end-labeling (TUNEL) assay. Labeled cells were detected by flow cytometry.

### Caspase-3 activity assay

Cell lysates were prepared and the caspase-3 activity was measured according to the manufacturer's instruction (#BF-1100) (R&D Systems, Minneapolis, Min., USA). Briefly, total protein (250 µg) was added into a reaction mixture including the fluorogenic peptide substrate (100 µM DEVD-AFC) specific for caspase-3, incubated at 37°C for 2 h. Fluorescence intensity was assessed using a Fluorescence plate reader (Fluoroskan Ascent; Labsystems, Helsinki, Finland) by exciting at 405 nm and emitting at 510 nm.

The article "Pemetrexed Induces S-Phase Arrest and Apoptosis via a Deregulated Activation of Akt Signaling Pathway" was retracted in 2024. Reasons: duplicated images; duplicated data; duplicate publication; overlap with earlier publications.

### Immunoprecipitation and Cdk2 kinase activity assay

In vitro Cdk2 kinase activity assay using histone H1 as the substrate was performed by a non-radioactive assay. Briefly, 300 µg of protein lysates from each sample was precleared with protein A/G-sepharose beads, and then anti-human Cdk2 antibody was mixed with cell lysates in the presence of 20 µl of protein G-sepharose beads, rotating at 4°C overnight. After washing with kinase reaction buffer, the histone H1 kinase activity of the immunocomplex was determined by incubation in 30 µl of kinase buffer [25 mM Tris-HCl pH 7.5, 5 mM β-glycerophosphate, 0.5 mM DTT, 0.1 mM Na_3_VO_4_, 20 mM MgCl_2_ and a serine/threonine phosphatase inhibitor cocktail (#20-201) (Merck Millipore, Billerica, MA., USA), 200 µM ATP, 0.5 mg/ml histone H1]. The kinase reaction was performed at 30°C for 45 minutes. The reaction was terminated by the addition of 10 µl of 4 x Laemmli sample buffer followed by boiling for 10 min. The end products were resolved on 12% SDS-polyacrylamide gel and detected by immunoblotting with phosphorylated histone H1 antibody.

### Immunofluorescence

Cells were seeded onto coverslips, treated with or without pemetrexed for the indicated period, and then cells were harvested and washed three times with PBS, fixed with 4% paraformaldehyde for 30 min at room temperature and permeabilized with 0.5% Triton X-100 for 30 min. After blocking in 1% bovine serum albumin, cells were incubated with an antibody against phospho-Akt^S473^ at 37°C for 1 h. Cells were then washed three times with PBS and detected with rhodamine-conjugated secondary antibodies. Hoechst 33342 was used to visualize cell nuclei. Cells were observed and photographed by confocal microscopy (FV1000) (Olympus, Tokyo, Japan).

### siRNA transfection

For siRNA transfection experiments, cells were plated onto 6 well (2×10^5^ per well) plates overnight, and then transiently transfected with Lipofectamine 2000 (#11668027) (Life Technology, Carlsbad, CA., USA) supplemented with Akt siRNA (10 and 25 nM). At 16 h post-transfection, cells were incubated without or with pemetrexed for the indicated time period. Subsequently, cells were collected for detection of the expressed levels of Akt protein by immunoblotting.

The article "Pemetrexed Induces S-Phase Arrest and Apoptosis via a Deregulated Activation of Akt Signaling Pathway" was retracted in 2024. Reasons: duplicated images; duplicated data; duplicate publication; overlap with earlier publications.

### Statistical analysis

All data were presented as mean±S.D. from three separate experiments. Statistical differences were evaluated using the Student's t-test and considered significant at the *p<0.05, **p<0.01, or ***p<0.001 level. The figures shown in this study were representative from at least three independent experiments with similar pattern.

## Results

### Pemetrexed-mediated Akt activation is accompanied by S-phase arrest and apoptotic cell death

Growing evidence shows that an Akt activated pathway plays a key role in cell cycle G1 to S phase progression [23]. Previous studies demonstrated that pemetrexed induces an epidermal growth factor receptor-mediated activation of the Akt pathway [20], [24]. Our recent reports indicate that pemetrexed induces cell cycle S-phase arrest in human NSCLC A549 cells [21], [22]. To examine the status of Akt in pemetrexed-treated cells, human NSCLC A549 cells were treated with pemetrexed for various time points. After treatment, the amount of S-phase population and apoptotic cell were assessed, the total cellular protein extracts were prepared and analyzed for phospho-specific Akt (Ser^473^) and total Akt proteins by immunoblot assay. As shown in Fig. 1, the level of phosphorylated Akt was increased by the pemetrexed treatment in a time- (Fig. 1A) and dose-dependent (Fig. 1B) manner, whereas the level of total Akt was relatively unchanged after pemetrexed treatment, indicating that the phosphorylated Akt levels were not due to differences in the abundance of total Akt protein. We also examined the phosphorylation status of GSK-3β, a known substrate of Akt. Indeed, the phosphorylation of GSK-3β correlated directly with the Akt phosphorylation status, supporting the view that the Akt pathway is functionally activated. In the meantime, the ratio of S-phase population and apoptotic cells was also increased by pemetrexed treatment (Figs. 1A & 1B).

**Figure 1:** Activation of Akt pathway by pemetrexed. (A) Akt activation in a time course dependent manner. Human lung adenocarcinoma A549 cells were treated without or with 1 µM pemetrexed for 0, 4, 8, 12, 24, and 48 h, and then cell lysates were isolated. (B) Akt activation occurred in a concentration dependent manner. A549 cells were treated with 0, 0.1, 0.3 and 1 µM pemetrexed for 48 h. After treatment, the levels of total Akt, phosphorylated Akt, total GSK3β, and phosphorylated GSK3β were examined by Western blot analysis. β-Actin was used as an internal loading control. The proportion of S-phase population and apoptotic cells was determined as described in the Materials and Methods section.

The article "Pemetrexed Induces S-Phase Arrest and Apoptosis via a Deregulated Activation of Akt Signaling Pathway" was retracted in 2024. Reasons: duplicated images; duplicated data; duplicate publication; overlap with earlier publications.

### Activation of the Akt signaling pathway contributes to pemetrexed-mediated S-phase arrest and apoptosis

To characterize whether pemetrexed-induced Akt activation and biological events were PI_3_K-dependent, A549 cells were pretreated with the PI_3_K-specific inhibitors, wortmannin and Ly294002, the levels of phosphorylated Akt and GSK3β were examined. As shown in Fig. 2A, in the presence of PI_3_K inhibitors, the pemetrexed-stimulated Akt and GSK3β phosphorylated activation were greatly diminished. However, treatment with PI_3_K inhibitor alone showed no significant difference in comparison with untreated control cells (data not shown). These results demonstrated that the elevated phosphorylated Akt was likely dependent on PI_3_K activity.

**Figure 2:** PI_3_K inhibitors suppress pemetrexed-induced Akt and GSK3β activation, S-phase arrest, cell apoptosis and caspase-3 activation.A549 were pretreated with 10 µM Ly294002 or 3 µM wortmannin (inhibitors of PI_3_K/Akt) for 2 h, and then 1 µM pemetrexed was added. (A) the levels of Akt and GSK3β and (B) the cell cycle distribution were determined for 24 h after pemetrexed treatment. (C) Cell apoptosis and (D) the caspase-3 activity were examined after 72 h pemetrexed incubation. **P<0.01, ***P<0.001.

Next, the effect of wortmannin and Ly294002 on pemetrexed-mediated S-phase arrest and cell viability were investigated. Wortmannin and Ly294002 effectively decreased pemetrexed-mediated S-phase arrest (Fig. 2B), while treatment with these two inhibitors alone showed no significant difference in cell cycle distribution compared to untreated cells (data not shown). These data indicate that PI_3_K/Akt activation facilitates the progression of cells from G1 into S phase in A549 cells, and that inhibition of Akt activity by wortmannin and Ly294002 prevents S-phase entrance. PI_3_K/Akt activation has been shown to exhibit both pro-apoptotic and anti-apoptotic effects in a variety of cellular systems [16], [18], [25]–[27]. To define the role of activated Akt in pemetrexed-induced apoptosis, A549 cells were incubated with 1 µM pemetrexed in the presence or absence of wortmannin and Ly294002 for 48 h andapoptosis was determined by TUNEL assay and caspase-3 activation. Results showed that wortmannin and Ly294002 significantly reduced apoptotic cells (Fig. 2C) and caspase-3 activity (Fig. 2D) induced by pemetrexed. However, treatment with these two PI_3_K inhibitors alone did not affect the cell viability and caspase-3 activity in comparison with untreated control cultures (data not shown). Moreover, knockdown of Akt expression using Akt-specific siRNA reduced the level of Akt protein (Fig. 3A), and blocked pemetrexed-mediated S-phase arrest (Fig. 3B). Under these conditions, we also found that A549 cells were more resistant to pemetrexed as determined by quantifying the apoptotic cells (Fig. 3C) and caspase-3 activity (Fig. 3D). These results indicate that the sustained activation of Akt is responsible for cell cycle S-phase arrest and cell death signaling in pemetrexed-treated A549 cells.

The article "Pemetrexed Induces S-Phase Arrest and Apoptosis via a Deregulated Activation of Akt Signaling Pathway" was retracted in 2024. Reasons: duplicated images; duplicated data; duplicate publication; overlap with earlier publications.

**Figure 3:** Knockdown of Akt by siRNA diminishes pemetrexed-induced S-phase arrest and apoptosis. Cells were transfected with 10 and 25-specific siRNA or scrambled siRNA for 16 h, and then incubated with 1 µM pemetrexed for 24 h; (A) the expression levels of Akt, and (B) cell cycle distribution were examined. (C) Apoptotic cells and (D) caspase-3 activity were assessed after 72 h pemetrexed treatment. ***P<0.001.

### Akt translocates to the nucleus during pemetrexed-induced cell death

Akt is commonly considered as a survival and proliferation promoting kinase. In the presence of pemetrexed, however, sustained activated Akt acts as a pro-apoptotic molecule, as its inhibition significantly blocks the cell death pathways induced by pemetrexed. Previous reports have shown that constitutive activation and nuclear localization of Akt promotes apoptosis in the presence of several chemotherapeutic drugs and apoptin [27], [28]. To further characterize the proapoptotic properties of Akt, the effect of pemetrexed on the cellular distribution of phosphor-Akt^S473^ was examined. As shown in Fig. 4A, phosphor-Akt^S473^ localized mainly in the cytoplasm, but slightly dispersed in the nucleus of untreated A549 cells. After treatment with pemetrexed, phosphor-Akt^S473^ gradually translocated and accumulated in the nucleus in a concentration-dependent manner. Time course experiments revealed that upon pemetrexed treatment, the majority of Akt was translocated to the nucleus within 12 h (Fig. 4B), a time that clearly preceded induction of S-phase arrest and cell death. It continued to accumulate in the nucleus even after 48 h of treatment. The nuclear localization of Akt is dependent on the upstream activation of PI_3_K, as the inhibition of PI_3_K activity by Ly294002 and wortmannin diminished the nuclear localization of Akt induced by pemetrexed (Fig. 4C). These results indicated that pemetrexed triggered the sustained activation and prolonged nuclear translocation of Akt in A549 cells.

**Figure 4:** Akt translocates to the nucleus during pemetrexed-induced cell death. (A) A549 cells were treated with 0, 0.1, 0.3, and 1 µM pemetrexed for 48 h, and (B) A549 cells were treated with 1 µM pemetrexed for 0, 12, 24, and 48 h. After treatment, the subcellular distribution of p-Akt^S473^ was detected by confocal microscopy after immunostaining with anti-phospho-Akt^S473^ and Rhodamine-conjugated secondary antibody. Hoechst 33342 was used to counter stain nuclei, and the images were overlaid to determine the Akt localization within the cell. (C) Inhibiton of Akt activation by Ly294002 and wortmannin blocked Akt nuclear accumulation. A549 cells were pretreated with 10 µM Ly294002 or 3 µM wortmannin for 2 h, and then 1 µM pemetrexed was added for another 48 h. The subcellular distribution of p-Akt^S473^ was detected by immunocytochemistry.

The article "Pemetrexed Induces S-Phase Arrest and Apoptosis via a Deregulated Activation of Akt Signaling Pathway" was retracted in 2024. Reasons: duplicated images; duplicated data; duplicate publication; overlap with earlier publications.

### Inhibition of Akt inactivates Cdk2/Cyclin A-associated kinase activity

Our previous report demonstrated that pemetrexed-induced apoptosis was closely associated with S-phase accumulation, as well as sustained Cdk2/cyclin A-associated kinase activation in human non-small cell lung cancer A549 cells [21]. To measure the activation of Cdk2 kinase activity, the in vitro kinase assay with histone H1 as the substrate was performed. Cdk2 activity was elevated in the presence of pemetrexed as indicated by histone H1 phosphorylation (Fig. 5A). By coimmunoprecipitation, we next determined whether active Cdk2 was associated with Cyclin E or Cyclin A. As shown in Fig. 5A, Cyclin A- but not Cyclin E-associated Cdk2 showed enhanced phosphorylation of histone H1, suggesting that only Cyclin A/Cdk2 was activated in pemetrexed-treated cells.

**Figure 5:** Inhibition of Akt activation suppresses pemetrexed-induced Cdk2 activation. (A) Pemetrexed stimulates Cdk2/Cyclin A-associated kinase activity. A549 cells were treated with 0, 0.3, and 1 µM pemetrexed for 24 h, and then protein lysates were isolated. Total protein (500 µg) was incubated with anti-Cdk2 antibody for immunoprecipitation of a Cdk2 kinase complex. Recombinant histone H1 protein was used as a substrate for the Cdk2 kinase activity assay. The levels of immunoprecipitated Cdk2, Cyclin A and Cyclin E were determined by immunoblotting with anti-Cdk2, anti-Cyclin A and anti-Cyclin E antibodies. β-Actin was used as an internal loading control. (B) Pharmacological inhibition of Akt activity decreases Cdk2 activity in pemetrexed-treated cells. A549 cells pretreated with 10 µM Ly294002 or 3 µM wortmannin for 2 h, and then 1 µM pemetrexed was added for another 24 h. The Cdk2 kinase activity and protein level were examined as above mentioned. (C) Knock down Akt expression by Akt specific siRNA reduces Cdk2 kinase activity. A549 cells were transfected with 25 nM of Akt-specific siRNA or scrambled siRNA for 16 h, and then incubated with 1 µM pemetrexed for 24 h, the Cdk2 kinase activity and protein levels were examined as above mentioned.

It has been shown that Akt phosphorylates Cdk2 both in vitro and in vivo during cell cycle progression and apoptosis [28]. We next examined whether the increased Cdk2 activity during a pemetrexed-induced event was dependent on Akt activation. Fig. 5B showed that Cdk2 was activated only when the Akt pathway remained intact. Prevention of Akt activation by wortmannin and Ly294002, two pharmacological PI_3_K inhibitors, strongly reduced Cdk2 activity. However, the Cdk2 activity of wortmannin and Ly294002 treatment alone was not altered in comparison with untreated cells (data not shown). In addition, knockdown of Akt expression by siRNA significantly attenuated pemetrexed-induced Cdk2 activity (Fig. 5C). These results therefore suggest that pemetrexed-induced Cdk2 activation required an intact PI_3_K/Akt pathway.

The article "Pemetrexed Induces S-Phase Arrest and Apoptosis via a Deregulated Activation of Akt Signaling Pathway" was retracted in 2024. Reasons: duplicated images; duplicated data; duplicate publication; overlap with earlier publications.

### Pemetrexed-induced apoptosis was also through an Akt-Cdk2 activated axis in H1299 cells

Our previous study demonstrated that the antitumor activities of pemetrexed were mediated by induction of S-phase arrest and apoptosis in both A549 and H1299 cell lines [22]; we next expanded our study to include H1299 cells. Consistently, treatment with pemetrexed significantly stimulated the Akt and GSK3β activation (Fig. 6A) and Akt nuclear accumulation (Fig. 6B). This event was accompanied by Cdk2/Cyclin A-associated kinase activation (Fig. 6C). Moreover, wortamannin and Ly294002 diminished pemetrexed-mediated Cdk2 activation (Fig. 7A), S phase arrest (Fig. 7B), apoptosis (Fig. 7C) and caspase-3 activity (Fig. 7D) in H1299 cells. However, these cellular and molecular events were not affected by wortmannin and Ly294002 treatment alone when compared to untreated cells (data not shown). These results indicate that activation of Akt-Cdk2/Cyclin A axis was one of the mechanisms for pemetrexed-mediated anti-lung cancer effect.

**Figure 6:** Activation of Akt and Cdk2 are occurred in pemetrexed-treated H1299 cells. (A) Pemetrexed stimulates Akt pathway activation. H1299 cells were treated with 0, 0.1, 0.3 and 1 µM pemetrexed for 48 h. After treatment, the levels of total Akt, phosphorylated Akt, total GSK3β, and phosphorylated GSK3β were examined by Western blot analysis. β-Actin was used as an internal loading control. The proportion of S-phase population and apoptotic cells were determined as described in the Materials and Methods section. (B) Nuclear accumulation of Akt occurred in pemetrexed-treated H1299 cells. Cells were treated with 0, 0.1, 0.3, and 1 µM pemetrexed for 48 h, the subcellular distribution of p-Akt^S473^ was detected by confocal microscopy after immunostaining with anti-phospho-Akt^S473^. Hoechst 33342 was used to counterstain nuclei. (C) Pemetrexed activated Cdk2/Cyclin A-associated kinase in H1299cells. H1299 cells were treated with 0, 0.3, and 1 µM pemetrexed for 24 h, and then protein lysates were isolated. The Cdk2 kinase activity and the levels of Cdk2, Cyclin A and Cyclin E were determined.

The article "Pemetrexed Induces S-Phase Arrest and Apoptosis via a Deregulated Activation of Akt Signaling Pathway" was retracted in 2024. Reasons: duplicated images; duplicated data; duplicate publication; overlap with earlier publications.

**Figure 7:** Pharmacological inhibition of Akt reduced pemetrexed-mediated Cdk2 activation, S-phase arrest and apoptosis in H1299 cells. Cells were pre-treated with wortmannin or Ly294002 for 2 h, and then treated with 1 µM pemetrexed, (A) the Cdk2 kinase activity and protein level were examined and (B) cell cycle distribution analysis was performed after 24 h treatment; (C) apoptotic cells and (D) caspase-3 activity were estimated after 72 h pemetrexed administration.

## Discussion

Pemetrexed has been reported to induce the selective death of tumor cells derived from diverse tissues or organs, whereas it has low toxicity to nontransformed cells [29]. Several studies demonstrated that pemetrexed-induced apoptosis was closely related to S-phase accumulation in human cancer cells [30]–[32]. In advanced non-squamous non-small cell lung cancer, pemetrexed is approved and commonly used as maintenance therapy after first-line chemotherapy [5]. It is well documented that pemetrexed acts as a thymidylate synthase inhibitor that interrupts the synthesis of DNA in tumor cells, resulting in decreased growth and induced death of the tumor cells. Clinically, thymidylate synthase has been suggested as a predictive biomarker for pemetrexed treatment in NSCLC patients [33]. However, the thymidylate synthase gene ubiquitously exists in normal and cancer cells, meaning that it may not be used to extensively explain the responsiveness to pemetrexed. It is possible that there are existed other potential biomarkers which may predict pemetrexed response. In an attempt to clearly elucidate the mechanism of the tumoricidal activity of pemetrexed in NSCLC, we previously identified components of the ERK and ATM signaling pathways as toxic determinants of pemetrexed in NSCLC A549 and H1299 cell lines [21], [22]. In this study, we provide for the first time a molecular mechanism for the unexpected proapoptotic role of the PI_3_K/Akt pathway by demonstrating that pemetrexed stimulated activation and nuclear retention of Akt, Cdk2/cyclin A is activated downstream of Akt. The sustained activation of Akt and Cdk2/Cyclin A-associated kinase leads to S-phase arrest and apoptosis in human NSCLC cell lines.

AKT, also known as protein kinase B (PKB), is a proto-oncoprotein and the central downstream effector molecule of the PI_3_K pathway. It is activated by interaction with the PtdIns(3,4,5)P3 and subsequent phosphorylation at S473 and T308 sites mediated by PDK1 and PDK2. Activation of PI_3_K/Akt signaling pathway in cells can maintain cell survival through inhibition of apoptosis by targeting BAD, caspase-9, NF-κB and FKHRL1 [34]. Additionally, Akt controls cell cycle progression by directly or indirectly targeting p21^waf1^, p27^kip1^, cyclin D, c-Myc, and GSK-3β [23]. It has been reported that prolonged activation of Akt causes a G2-M phase cell cycle arrest [28], [35]. In contrast to the role of the Akt pathway in cell proliferation and cell survival, Akt has also been shown to be involved in promotion of cell death [15]–[17]. A previous study showed that unscheduled Akt activation leads to apoptosis [26]. Sustained activation of Akt induced by both methotrexate and docetaxel not only played a role in cell cycle arrest but also has a very crucial role in apoptosis in human breast cancer MCF7 cells [28]. Pemetrexed has been shown to induce an epidermal growth factor receptor-mediated activation of the PI_3_K/Akt pathway and S-phase block in A549 cells, which was inhibited by a specific PI_3_K, Ly294002 [20]. Besides, Li *et al*., demonstrated an increase of Akt-Ser473 by pemetrexed in both dose- and time-dependent manners in erlotinib-resistant A549 cells [20]. Moreover, Bischof *et al*., showed that the administration of pemetrexed to human dermal microvascular endothelial cells induced the phosphorylation of Akt-Ser473 [36]. In agreement with these studies, we found that prolonged Akt activation was accompanied by the S-phase arrest and apoptosis in pemetrexed-treated NSCLC cell lines. In contrast to its extensively documented antiapoptotic effect, the activated Akt appears to play a crucial role in pemetrexed-induced toxicity, as both pretreatment of cells with the pharmacological inhibitors (wortmannin and Ly294002) and knockdown Akt expression by Akt-specific siRNA significantly abrogated S-phase arrest and improved the survival of pemetrexed-treated A549 cells (Figs. 2 & 3). These results suggest that prolonged and continuous activation of Akt contributes to pemetrexed-induced S-phase arrest and apoptotic cell death. However, several studies showed conflicting results regarding the modulation of phospho-Akt levels by pemetrexed. The decrease of phospho-Akt levels may contribute to the increased apoptosis after pemetrexed treatment in human lung cancer A549 cells [24], [37] and in human malignant pleural mesothelioma cell lines [38]. The reason for the controversial findings in modulation of phospho-Akt by pemetrexed remains to be determined, but may relate to the discrepancy between drug exposure conditions and different sensitivities of experimental methods.

The article "Pemetrexed Induces S-Phase Arrest and Apoptosis via a Deregulated Activation of Akt Signaling Pathway" was retracted in 2024. Reasons: duplicated images; duplicated data; duplicate publication; overlap with earlier publications.

Cell cycle progression is controlled by a set of Cyclins/Cdks complexes, and their abnormal expression may play an important role in the pathogenesis of human cancers [39]. It is well known that Cdk2/Cyclin A complex plays a key role in DNA synthesis and S-phase progression [40], [41]. Increased expression of Cyclin A has been detected in many types of human cancers, which appears to be of prognostic values such as prediction of survival or early relapse [42]. It has been reported that the tumor tissue negativity for Cyclin A expression predicts a favorable outcome in human NSCLC [43]. Several studies suggest that increased gene expression and enhanced kinase activity of Cdk2/Cyclin A plays an essential role in S-phase arrest and/or apoptosis [44]-[46]. Cdk2 activity has been shown to be selectively up-regulated and that this up-regulation is required for the induction of apoptosis by ginsenoside Rh2 [47], panaxadiol [48], and etoposide [49] in various cancer cell lines. Our previous study provided strong evidence that ERK1/2-dependent Cdk2/Cyclin A-associated kinase activation is an important mediator of pemetrexed-induced S-phase arrest and apoptosis [21]. This study showed that pemetrexed-induced Cdk2/Cyclin A activation was PI_3_K/Akt signaling pathway dependent. Using the PI_3_K inhibitors (Ly294002 and wortamanin) as well as small interference RNA knockdown Akt expression resulted in a loss of Cdk2/Cyclin A expression and kinase activity (Figs. 2A & 3A), and significantly decreased S-phase arrest (Figs. 2B & 3B) and cell death (Figs. 2C & 3C) upon pemetrexed treatment. Similarly, Eapen *et al*. Showed that cytokines stimulate Cdk2 activation through a PI_3_K/Akt-dependent signaling pathway and promote cell cycle progression during γ-IR-induced DNA damage in hematopoietic cells [50]. Another report demonstrated that erythropoietin and interleukin-3 activate a PI_3_K/Akt-Cdk1/2 signaling pathway; this signaling axis can override cisplatin-induced growth arrest checkpoints, thereby sensitizing hematopoietic cells to DNA damage-induced death [17]. Maddika *et al.* reported that Cdk2 is a novel target for Akt and has a role not only during cell cycle progression but also during apoptosis [27], [28]. These findings suggest that Cyclin A-Cdk2 regulated cell cycle arrest and apoptosis are PI_3_K/Akt dependent.

In this study, the downstream targets for Cdk2/Cyclin A during S-phase arrest and cell death induced by pemetrexed have not yet been clarified. Cdk2/Cyclin A has been shown to act upstream of mitochondrial cytochrome c release in the apoptosis pathway [45], [47]. A recent report indicated that sustained activation of Cyclin A-Cdk2 triggers Rad9 phosphorylation and thereby promotes the interaction of Rad9 with Bcl-xL and the subsequent initiation of the apoptotic program in HeLa cells [46]. Our previous study showed that pemetrexed-induced both death receptor- and mitochondria-dependent apoptosis in A549 cells. Whether Cyclin A-Cdk2-mediated Rad9 phosphorylation and interaction with Bcl-xL is another mechanism involved in pemetrexed-induced cell death needs to be explored. Further identification of additional Cdk2/Cyclin A targets might provide clues about the different roles of Cdk2/Cyclin A in cell cycle progression and apoptosis.

The article "Pemetrexed Induces S-Phase Arrest and Apoptosis via a Deregulated Activation of Akt Signaling Pathway" was retracted in 2024. Reasons: duplicated images; duplicated data; duplicate publication; overlap with earlier publications.

Growing evidence strongly suggests that nuclear-cytoplasmic shuttling of certain pro-apoptotic kinases, including PKCδ[51]-[53], DYRK2 [54] and c-Abl [55], [56] is essential for induction of apoptosis in response to DNA damage or various cell-death stimuli. Interestingly, here we showed that Akt was sustained activated and accumulated in the nucleus during pemetrexed treatment and that this was required for its S-phase arrest and cell-death inducing activities (Figs. 4, 5, & 6). This result is consistent with the finding that the nuclear translocation and activation of Akt, resulting in the subsequent phosphorylation and activation of Cdk2, is required for apoptin-induced apoptosis [27], [57]. Akt is predominantly expressed in the cytoplasm. Maddika *et al* demonstrated that activated Akt may translocate to the nucleus during the S phase and may phosphorylate Cdk2 and promote cytoplasmic Cdk2 localization during late S and G2 phases of the normal cell cycle. In addition to their role in cell cycle progression, the Akt/Cdk2 pathway has been also shown to promote apoptosis in response to several death-inducing stimuli, including methotrexate and docetaxel [28]. These results reveal that transient and cell-cycle regulated activation of Akt and shuttling between the nucleus and the cytoplasm is characteristic for normal activation by pro-survival pathways during cell cycle progression [28]. Conversely, prolonged activation and nuclear accumulation of Akt promotes apoptosis. These findings indicate that sustained activation of Akt/Cdk2 and aberrant subcellular distribution might contribute to the induction of cell cycle arrest and/or cell death of these kinases. Importantly, Akt has no nuclear localization signal. It may require additional nuclear targeting partners for its nuclear translocation, whereas precise regulation for the nucleus-cytoplasm shuttling of Akt remains unclear and needs to be further explored.

Our previous reports indicated that pemetrexed induced the apoptosis of A549 (wild-type p53) and H1299 (p53 null) lung cancer cell lines [21], [22], suggesting that p53 is important but not necessary for pemetrexed-induced cell death. The present study further showed that pemetrexed-induced S-phase arrest and apoptosis were via the activation of Akt-Cdk2 axis in both A549 and H1299 cell lines. Our findings clearly indicate that the pemetrexed-induced signaling pathways and antitumor effects in lung cancer cells are through both p53-dependent and p53-independent pathways.

The article "Pemetrexed Induces S-Phase Arrest and Apoptosis via a Deregulated Activation of Akt Signaling Pathway" was retracted in 2024. Reasons: duplicated images; duplicated data; duplicate publication; overlap with earlier publications.

In conclusion, our results show for the first time that the sustained activation and nuclear accumulation of Akt contribute to pemetrexed-induced S-phase arrest and apoptosis in human NSCLC A549 and H1299 cell lines. Akt activation stimulated Cdk2/Cyclin A-associated kinase activation and then promoted the movement of cells into the S phase, and prolonged and unscheduled activation of Akt and Cdk2/Cyclin-A might create a cellular disharmony which eventually led to apoptosis (Fig. 8). Due to pemetrexed having a lower cytotoxicity to normal cells, our findings may have clinical relevance considering the fact that tumor cells usually have overexpressed Cyclin-A, Cdks, and Akt activity [42], [58]–[60]. The clinical efficacy of pemetrexed in the treatment of patients with non-small cell lung cancer, especially those with high Akt kinase activity and Cdk2/Cyclin-A expression, is worthy of further investigation.

**Figure 8:** Schematic representation of the molecular mechanisms of pemetrexed-induced growth arrest and cell death in human NSCLC cell lines.

## References

[1] LeeYC, WuCT, ChenCS, HsuHH, ChangYL (2002) The significance of E-cadherin and alpha-, beta-, and gamma-catenin expression in surgically treated non-small cell lung cancers of 3 cm or less in size. J Thorac Cardiovasc Surg 123: 502–507.1188282210.1067/mtc.2002.119334

[2] WakeleeH, BelaniCP (2005) Optimizing first-line treatment options for patients with advanced NSCLC. Oncologist 10 Suppl 31–10.10.1634/theoncologist.10-90003-116368866

[3] RamalingamS, BelaniC (2008) Systemic chemotherapy for advanced non-small cell lung cancer: recent advances and future directions. Oncologist 13 Suppl 15–13.1826376910.1634/theoncologist.13-S1-5

[4] EdelmanMJ, Le ChevalierT, SoriaJC (2012) Maintenance therapy and advanced non-small-cell lung cancer: a skeptic's view. J Thorac Oncol 7: 1331–1336.2289513710.1097/JTO.0b013e3182629e37

[5] GreenhalghJ, McLeodC, BagustA, BolandA, FleemanN, et al (2010) Pemetrexed for the maintenance treatment of locally advanced or metastatic non-small cell lung cancer. Health Technol Assess 14: 33–39.2104748910.3310/hta14suppl2/05

[6] GonenN, AssarafYG (2012) Antifolates in cancer therapy: structure, activity and mechanisms of drug resistance. Drug Resist Updat 15: 183–210.2292131810.1016/j.drup.2012.07.002

The article "Pemetrexed Induces S-Phase Arrest and Apoptosis via a Deregulated Activation of Akt Signaling Pathway" was retracted in 2024. Reasons: duplicated images; duplicated data; duplicate publication; overlap with earlier publications.

[7] BrittenCD, IzbickaE, HilsenbeckS, LawrenceR, DavidsonK, et al (1999) Activity of the multitargeted antifolate LY231514 in the human tumor cloning assay. Cancer Chemother Pharmacol 44: 105–110.1041294310.1007/s002800050953

[8] TeicherBA, AlvarezE, LiuP, LuK, MenonK, et al (1999) MTA (LY231514) in combination treatment regimens using human tumor xenografts and the EMT-6 murine mammary carcinoma. Semin Oncol 26: 55–62.10598556

[9] TeicherBA, ChenV, ShihC, MenonK, ForlerPA, et al (2000) Treatment regimens including the multitargeted antifolate LY231514 in human tumor xenografts. Clin Cancer Res 6: 1016–1023.10741729

[10] VadlakondaL, DashA, PasupuletiM, Anil KumarK, ReddannaP (2013) The Paradox of Akt-mTOR Interactions. Front Oncol 3: 165.2380209910.3389/fonc.2013.00165PMC3687210

[11] VadlakondaL, PasupuletiM, PalluR (2013) Role of PI3K-AKT-mTOR and Wnt Signaling Pathways in Transition of G1-S Phase of Cell Cycle in Cancer Cells. Front Oncol 3: 85.2359656910.3389/fonc.2013.00085PMC3624606

[12] WelkerME, KulikG (2013) Recent syntheses of PI3K/Akt/mTOR signaling pathway inhibitors. Bioorg Med Chem 21: 4063–4091.2373583110.1016/j.bmc.2013.04.083PMC3711139

[13] MaX, HuY (2013) Targeting PI3K/Akt/mTOR cascade: the medicinal potential, updated research highlights and challenges ahead. Curr Med Chem 20: 2991–3010.2365130310.2174/09298673113209990124

[14] KhanKH, YapTA, YanL, CunninghamD (2013) Targeting the PI3K-AKT-mTOR signaling network in cancer. Chin J Cancer 32: 253–265.2364290710.5732/cjc.013.10057PMC3845556

[15] AkiT, YamaguchiK, FujimiyaT, MizukamiY (2003) Phosphoinositide 3-kinase accelerates autophagic cell death during glucose deprivation in the rat cardiomyocyte-derived cell line H9c2. Oncogene 22: 8529–8535.1462799410.1038/sj.onc.1207197

[16] LuB, WangL, StehlikC, MedanD, HuangC, et al (2006) Phosphatidylinositol 3-kinase/Akt positively regulates Fas (CD95)-mediated apoptosis in epidermal Cl41 cells. J Immunol 176: 6785–6793.1670983810.4049/jimmunol.176.11.6785

[17] NimbalkarD, HenryMK, QuelleFW (2003) Cytokine activation of phosphoinositide 3-kinase sensitizes hematopoietic cells to cisplatin-induced death. Cancer Res 63: 1034–1039.12615719

[18] ShackS, WangXT, KokkonenGC, GorospeM, LongoDL, et al (2003) Caveolin-induced activation of the phosphatidylinositol 3-kinase/Akt pathway increases arsenite cytotoxicity. Mol Cell Biol 23: 2407–2414.1264012410.1128/MCB.23.7.2407-2414.2003PMC150728

[19] NarayanRS, FedrigoCA, StalpersLJ, BaumertBG, SminiaP (2013) Targeting the Akt-pathway to improve radiosensitivity in glioblastoma. Curr Pharm Des 19: 951–957.22973963

[20] LiT, LingYH, GoldmanID, Perez-SolerR (2007) Schedule-dependent cytotoxic synergism of pemetrexed and erlotinib in human non-small cell lung cancer cells. Clin Cancer Res 13: 3413–3422.1754555010.1158/1078-0432.CCR-06-2923

The article "Pemetrexed Induces S-Phase Arrest and Apoptosis via a Deregulated Activation of Akt Signaling Pathway" was retracted in 2024. Reasons: duplicated images; duplicated data; duplicate publication; overlap with earlier publications.

[21] YangTY, ChangGC, ChenKC, HungHW, HsuKH, et al (2011) Sustained activation of ERK and Cdk2/cyclin-A signaling pathway by pemetrexed leading to S-phase arrest and apoptosis in human non-small cell lung cancer A549 cells. Eur J Pharmacol 663: 17–26.2157563110.1016/j.ejphar.2011.04.057

[22] YangTY, ChangGC, ChenKC, HungHW, HsuKH, et al (2013) Pemetrexed induces both intrinsic and extrinsic apoptosis through ataxia telangiectasia mutated/p53-dependent and -independent signaling pathways. Mol Carcinog 52: 183–194.2208665810.1002/mc.21842

[23] LiangJ, SlingerlandJM (2003) Multiple roles of the PI3K/PKB (Akt) pathway in cell cycle progression. Cell Cycle 2: 339–345.12851486

[24] TekleC, GiovannettiE, SigmondJ, GraffJR, SmidK, et al (2008) Molecular pathways involved in the synergistic interaction of the PKC beta inhibitor enzastaurin with the antifolate pemetrexed in non-small cell lung cancer cells. Br J Cancer 99: 750–759.1872866610.1038/sj.bjc.6604566PMC2528136

[25] StilesBL (2009) PI-3-K and AKT: Onto the mitochondria. Adv Drug Deliv Rev 61: 1276–1282.1972009910.1016/j.addr.2009.07.017

[26] van GorpAG, PomeranzKM, BirkenkampKU, HuiRC, LamEW, et al (2006) Chronic protein kinase B (PKB/c-akt) activation leads to apoptosis induced by oxidative stress-mediated Foxo3a transcriptional up-regulation. Cancer Res 66: 10760–10769.1710811210.1158/0008-5472.CAN-06-1111

[27] MaddikaS, PanigrahiS, WiechecE, WesselborgS, FischerU, et al (2009) Unscheduled Akt-triggered activation of cyclin-dependent kinase 2 as a key effector mechanism of apoptin's anticancer toxicity. Mol Cell Biol 29: 1235–1248.1910374210.1128/MCB.00668-08PMC2643822

[28] MaddikaS, AndeSR, WiechecE, HansenLL, WesselborgS, et al (2008) Akt-mediated phosphorylation of CDK2 regulates its dual role in cell cycle progression and apoptosis. J Cell Sci 121: 979–988.1835408410.1242/jcs.009530PMC2954964

[29] WelshSJ, TitleyJ, BruntonL, ValentiM, MonaghanP, et al (2000) Comparison of thymidylate synthase (TS) protein up-regulation after exposure to TS inhibitors in normal and tumor cell lines and tissues. Clin Cancer Res 6: 2538–2546.10873110

[30] TonkinsonJL, MarderP, AndisSL, SchultzRM, GossettLS, et al (1997) Cell cycle effects of antifolate antimetabolites: implications for cytotoxicity and cytostasis. Cancer Chemother Pharmacol 39: 521–531.911846410.1007/s002800050608

[31] JacksonRC (1984) Biological effects of folic acid antagonists with antineoplastic activity. Pharmacol Ther 25: 61–82.638772510.1016/0163-7258(84)90024-x

The article "Pemetrexed Induces S-Phase Arrest and Apoptosis via a Deregulated Activation of Akt Signaling Pathway" was retracted in 2024. Reasons: duplicated images; duplicated data; duplicate publication; overlap with earlier publications.

[32] TonkinsonJL, WorzallaJF, TengCH, MendelsohnLG (1999) Cell cycle modulation by a multitargeted antifolate, LY231514, increases the cytotoxicity and antitumor activity of gemcitabine in HT29 colon carcinoma. Cancer Res 59: 3671–3676.10446980

[33] TakezawaK, OkamotoI, OkamotoW, TakedaM, SakaiK, et al (2011) Thymidylate synthase as a determinant of pemetrexed sensitivity in non-small cell lung cancer. Br J Cancer 104: 1594–1601.2148740610.1038/bjc.2011.129PMC3101907

[34] CantleyLC (2002) The phosphoinositide 3-kinase pathway. Science 296: 1655–1657.1204018610.1126/science.296.5573.1655

[35] AlvarezB, MartinezAC, BurgeringBM, CarreraAC (2001) Forkhead transcription factors contribute to execution of the mitotic programme in mammals. Nature 413: 744–747.1160703410.1038/35099574

[36] BischofM, AbdollahiA, GongP, StoffregenC, LipsonKE, et al (2004) Triple combination of irradiation, chemotherapy (pemetrexed), and VEGFR inhibition (SU5416) in human endothelial and tumor cells. Int J Radiat Oncol Biol Phys 60: 1220–1232.1551979510.1016/j.ijrobp.2004.07.689

[37] GiovannettiE, MeyV, NannizziS, PasqualettiG, MariniL, et al (2005) Cellular and pharmacogenetics foundation of synergistic interaction of pemetrexed and gemcitabine in human non-small-cell lung cancer cells. Mol Pharmacol 68: 110–118.1579532010.1124/mol.104.009373

[38] GiovannettiE, ZucaliPA, AssarafYG, LeonLG, SmidK, et al (2011) Preclinical emergence of vandetanib as a potent antitumour agent in mesothelioma: molecular mechanisms underlying its synergistic interaction with pemetrexed and carboplatin. Br J Cancer 105: 1542–1553.2197087410.1038/bjc.2011.400PMC3242521

[39] GranaX, ReddyEP (1995) Cell cycle control in mammalian cells: role of cyclins, cyclin dependent kinases (CDKs), growth suppressor genes and cyclin-dependent kinase inhibitors (CKIs). Oncogene 11: 211–219.7624138

[40] HuangX, SummersMK, PhamV, LillJR, LiuJ, et al (2011) Deubiquitinase USP37 is activated by CDK2 to antagonize APC(CDH1) and promote S phase entry. Mol Cell 42: 511–523.2159631510.1016/j.molcel.2011.03.027

[41] NeganovaI, VilellaF, AtkinsonSP, LloretM, PassosJF, et al (2011) An important role for CDK2 in G1 to S checkpoint activation and DNA damage response in human embryonic stem cells. Stem Cells 29: 651–659.2131927310.1002/stem.620

[42] YamCH, FungTK, PoonRY (2002) Cyclin A in cell cycle control and cancer. Cell Mol Life Sci 59: 1317–1326.1236303510.1007/s00018-002-8510-yPMC11337442

[43] VolmM, RittgenW, DringsP (1998) Prognostic value of ERBB-1, VEGF, cyclin A, FOS, JUN and MYC in patients with squamous cell lung carcinomas. Br J Cancer 77: 663–669.948482710.1038/bjc.1998.106PMC2149928

[44] AdachiS, ItoH, Tamamori-AdachiM, OnoY, NozatoT, et al (2001) Cyclin A/cdk2 activation is involved in hypoxia-induced apoptosis in cardiomyocytes. Circ Res 88: 408–414.1123010810.1161/01.res.88.4.408

The article "Pemetrexed Induces S-Phase Arrest and Apoptosis via a Deregulated Activation of Akt Signaling Pathway" was retracted in 2024. Reasons: duplicated images; duplicated data; duplicate publication; overlap with earlier publications.

[45] DingH, HanC, GuoD, WangD, ChenCS, et al (2008) OSU03012 activates Erk1/2 and Cdks leading to the accumulation of cells in the S-phase and apoptosis. Int J Cancer 123: 2923–2930.1879825710.1002/ijc.23896

[46] ZhanZ, HeK, ZhuD, JiangD, HuangYH, et al (2012) Phosphorylation of Rad9 at serine 328 by cyclin A-Cdk2 triggers apoptosis via interfering Bcl-xL. PLoS One 7: e44923.2302868210.1371/journal.pone.0044923PMC3441668

[47] JinYH, YooKJ, LeeYH, LeeSK (2000) Caspase 3-mediated cleavage of p21WAF1/CIP1 associated with the cyclin A-cyclin-dependent kinase 2 complex is a prerequisite for apoptosis in SK-HEP-1 cells. J Biol Chem 275: 30256–30263.1088438210.1074/jbc.M001902200

[48] JinYH, YimH, ParkJH, LeeSK (2003) Cdk2 activity is associated with depolarization of mitochondrial membrane potential during apoptosis. Biochem Biophys Res Commun 305: 974–980.1276792610.1016/s0006-291x(03)00870-2

[49] ChoiJS, ShinS, JinYH, YimH, KooKT, et al (2007) Cyclin-dependent protein kinase 2 activity is required for mitochondrial translocation of Bax and disruption of mitochondrial transmembrane potential during etoposide-induced apoptosis. Apoptosis 12: 1229–1241.1725219510.1007/s10495-006-0047-3

[50] EapenAK, HenryMK, QuelleDE, QuelleFW (2001) Dna damage-induced G(1) arrest in hematopoietic cells is overridden following phosphatidylinositol 3-kinase-dependent activation of cyclin-dependent kinase 2. Mol Cell Biol 21: 6113–6121.1150965410.1128/MCB.21.18.6113-6121.2001PMC87328

[51] YoshidaK, WangHG, MikiY, KufeD (2003) Protein kinase Cdelta is responsible for constitutive and DNA damage-induced phosphorylation of Rad9. EMBO J 22: 1431–1441.1262893510.1093/emboj/cdg134PMC151076

[52] EitelK, StaigerH, RiegerJ, MischakH, BrandhorstH, et al (2003) Protein kinase C delta activation and translocation to the nucleus are required for fatty acid-induced apoptosis of insulin-secreting cells. Diabetes 52: 991–997.1266347110.2337/diabetes.52.4.991

[53] DeVries-SeimonTA, OhmAM, HumphriesMJ, ReylandME (2007) Induction of apoptosis is driven by nuclear retention of protein kinase C delta. J Biol Chem 282: 22307–22314.1756270710.1074/jbc.M703661200

[54] TairaN, NihiraK, YamaguchiT, MikiY, YoshidaK (2007) DYRK2 is targeted to the nucleus and controls p53 via Ser46 phosphorylation in the apoptotic response to DNA damage. Mol Cell 25: 725–738.1734995810.1016/j.molcel.2007.02.007

[55] YoshidaK, YamaguchiT, NatsumeT, KufeD, MikiY (2005) JNK phosphorylation of 14-3-3 proteins regulates nuclear targeting of c-Abl in the apoptotic response to DNA damage. Nat Cell Biol 7: 278–285.1569615910.1038/ncb1228

The article "Pemetrexed Induces S-Phase Arrest and Apoptosis via a Deregulated Activation of Akt Signaling Pathway" was retracted in 2024. Reasons: duplicated images; duplicated data; duplicate publication; overlap with earlier publications.

[56] RainaD, AhmadR, KumarS, RenJ, YoshidaK, et al (2006) MUC1 oncoprotein blocks nuclear targeting of c-Abl in the apoptotic response to DNA damage. EMBO J 25: 3774–3783.1688862310.1038/sj.emboj.7601263PMC1553184

[57] MaddikaS, BayGH, KroczakTJ, AndeSR, MaddikaS, et al (2007) Akt is transferred to the nucleus of cells treated with apoptin, and it participates in apoptin-induced cell death. Cell Prolif 40: 835–848.1802117410.1111/j.1365-2184.2007.00475.xPMC2954966

[58] DaiY, GrantS (2003) Cyclin-dependent kinase inhibitors. Curr Opin Pharmacol 3: 362–370.1290194410.1016/s1471-4892(03)00079-1

[59] SchuurbiersOC, KaandersJH, van der HeijdenHF, DekhuijzenRP, OyenWJ, et al (2009) The PI3-K/AKT-pathway and radiation resistance mechanisms in non-small cell lung cancer. J Thorac Oncol 4: 761–767.1940421810.1097/JTO.0b013e3181a1084f

[60] GadgeelSM, WozniakA (2013) Preclinical rationale for PI3K/Akt/mTOR pathway inhibitors as therapy for epidermal growth factor receptor inhibitor-resistant non-small-cell lung cancer. Clin Lung Cancer 14: 322–332.2333228710.1016/j.cllc.2012.12.001

